The article "Logistic Model and Gradient Boosting Machine Model for Physical Therapy of Lumbar Disc Herniation" was published in 2022. Journal: Comput Math Methods Med.

# Logistic Model and Gradient Boosting Machine Model for Physical Therapy of Lumbar Disc Herniation

**DOI:** 10.1155/2022/4799248

**Published:** 2022-05-11

**Authors:** Ping Zhao, Jin Xue, Xiaomei Xu, Lifei Wang, Dan Chen

**Affiliations:** ^1^Nursing Department, The Third People's Hospital of Hefei, Hefei Third Clinical College of Anhui Medical University, Hefei 230022, China; ^2^Department of Orthopaedics, The Third People's Hospital of Hefei, Hefei Third Clinical College of Anhui Medical University, Hefei 230022, China; ^3^Department of Neurosurgery, The Third People's Hospital of Hefei, Hefei Third Clinical College of Anhui Medical University, Hefei 230022, China

## Abstract

**Objective:**

Physical therapy is a common clinical treatment for patients with lumbar disc herniation. The study is aimed at exploring the feasibility of mathematical expression and curative effect prediction of physical therapy in patients with lumbar disc herniation using a logistic model and gradient boosting machine (GBM).

**Methods:**

A total of 142 patients with lumbar disc herniation were treated with physical therapy. The pain was evaluated by the visual analogue scale (VAS) before each treatment. The logistic model was used to conduct a global regression analysis on patients with lumbar disc herniation. The final results of the whole course of treatment were predicted by the measured values of 2-9 times of treatment. The GBM model was used to predict and analyze the curative effect of physical therapy.

**Results:**

The mathematical expression ability of the logistic regression model for patients with lumbar disc herniation undergoing physical therapy was sufficient, and the global determination coefficient was 0.721. The results would be better for more than five measurements. The AUC of GBM mode logistic regression analysis was 0.936 and 0.883, and the prediction effect is statistically significant.

**Conclusion:**

Both the logistic and GBM model can fully express the changes in patients with lumbar disc herniation during physical therapy.

## 1. Introduction

Lumbar disc herniation, the most common degenerative spine disease, can cause low back pain and sciatica, causing great distress to patients' daily life [1]. Timely physical treatment can achieve traction disc, joint loosening, and other effects to relieve the patient's lumbar pain and sciatica. Physical therapy has many advantages, such as easy and reliable efficacy. Thus, it is widely used in the clinic and plays an important therapeutic role [2]. In clinical rehabilitation practice, how to optimize the prescription and further improve the efficacy is one of the important topics of concern for clinical rehabilitation workers. There are numerous reports on analyzing rehabilitation efficacy in lumbar disc herniation. However, due to interindividual variability and the diversity of physical therapy, physical therapy prescriptions often have distinct individualized characteristics, which also poses some difficulties for efficacy prediction [3]. In clinical practice, predicting efficacy by an investigational treatment is widely adopted. In this process, three aspects have become the key to optimizing the configuration of medical resources and improving the efficiency of rehabilitation treatment: how to determine the appropriate length of treatment time, accurately estimate the efficacy of the entire course of therapy; timely termination of the treatment regimens that may be less effective [4–9].

Machine learning is a multidomain interdisciplinary emerging over the last 20 years, involving several disciplines such as probability theory, statistics, approximation, convex analysis, and algorithmic complexity theory [10–14]. It is an essential branch of computer science mainly used to model complex relationships between predictor and response variables and has the potential to transform modern methods of epidemiological research. With “big data” attracting much attention, machine learning can provide epidemiologists with new tools and ideas for solving problems that traditional methods cannot solve [15]. The gradient boosting machine (GBM), a machine learning algorithm for regression and classification, can train many models in order. Then, each new model updates the prediction using the gradient descent method [16–20]. GBM has shown great success in a wide range of practical applications and can be highly customized to the application's specific needs, gradually minimizing the loss of function. The logistic regression model is a classical linear regression model that can mine the linear relationship before variables and establish an effective model to predict future variable results.

The logistic curve model was used for the mathematical expression on the treatment process of cervical radicular pain. The prediction of the effect of physical therapy on cervical radicular pain was achieved by further mathematical feature analysis and predictive ability analysis [21–23]. During physical therapy, patients with cervical spondylosis show a closer course of remission than patients with lumbar disc herniation. Based on the above background, this study attempted to apply the GBM model and logistic model to describe the process of physical therapy and the prediction of efficacy in patients with lumbar disc herniation.

## 2. Material and Method

### 2.1. General Data

A total of 142 patients with lumbar disc herniation, aged 17 to 87 years (53.1 ± 15.2) years, who were treated at the Department of physical medicine and rehabilitation of our hospital from December 2018 to June 2021, were selected, including 89 males and 53 females. Inclusion criteria were as follows: (1) they met the diagnostic criteria of lumbar disc herniation according to the diagnosis and treatment code of China Rehabilitation Medicine based on the symptom presentation, physical examination, and auxiliary examinations, accompanied by radicular radiation pain; (2) they can understand and apply visual analog scale for pain rating; (3) they can adhere to completion of more than ten physical therapy sessions; (4) the patient's condition was stable.

The patient after admission determined the corresponding physical therapy prescription according to his actual condition. The treatment contents included traction, joint loosening, and physical factor therapy. These treatments were used once daily for five consecutive days each week, ten times for one course. The visual analogue scale (VAS) pain assessment was performed simultaneously before each treatment. The specific method is to draw a 10 cm long line segment in front of the patient and inform the patient that the left end of the line segment represents no pain, and the right end of the line segment represents intolerable severe pain and asked patients to label the average degree of pain in the past 24 h on the line segment. The researcher then used a ruler to measure the distance from the left endpoint of the line segment to the marked point and recorded each patient to the end of the course to obtain ten pain VAS score values. Throughout treatment, every effort was made to guarantee that each patient's treatment time point was relatively fixed.

### 2.2. Mathematical Expression and Predictive Power Analysis

Using the logistic model as a regression analysis model, *y* represents the degree of pain during treatment, and *x* represents the time point to complete treatment. The corresponding *x* values at the 10 measurement time points in this study are 1, 2,…, 9, 10. The *a*, *b* is the parameter, and the *H* is the distance between the upper and lower asymptotes representing the maximum possible relief during treatment as determined by the pain level at the initial visit. According to the vas minimal clinically significant difference (MCSD) theory proposed by Kelly [24], the position of the upper asymptote is defined as the level 1.2 above the 1st pain score value, i.e., *K* value = 1st VAS + 1.2. Since the maximum value of the VAS score is 10, the *K* value was taken as 10 when the VAS ≥ 8.8 at the first assessment.

To explore the predictive ability of different treatment duration, the predictive models were constructed with the measurement results of 1st to 2nd, 1st to 3rd, 1st to 4th, 1st to 5th, 1st to 6th, 1st to 7th, 1st to 8th, and 1st to 9th. The logistic model curve fitting analysis were completed. The predicted value of each model for the degree of pain at the 10th rating time point was then evaluated, and the difference between this expected value and the actual measurement was calculated.

Based on the actual measured values and MCSD theory, cases with a decrease of more than 1.2 VAS score on the whole course were defined as clinically effective cases, and the cases with less than 1.2 points were defined as invalid cases. The magnitude of decline predicted by each model was calculated simultaneously, and cases with a decrease of more than 1.2 points were defined as predicted valid cases. Cases with a decrease of less than 1.2 points were defined as predicted null cases. When the expected outcome was consistent with the actual measured outcome, it was defined as the predicted successful case and vice versa as the expected unsuccessful case. The predictive ability of different predictive models was compared between groups.

Remission magnitude was defined as predicting a successful case and vice versa an unsuccessful case when the difference between the predicted value and the actual measured last score value was within 1.2 points. The success rate predicted by the remission magnitude was calculated for each length of treatment, and the difference between the models in predicting remission magnitude was compared.

### 2.3. GBM Model Construction

Data acquisition, data preprocessing, training, model evaluation, and prediction for GBM models were implemented using Python 3.8 (https://www.python.org/downloads/Guido van Rossum). The data were randomly divided into training and test sets in a 7 : 3 ratio, and the optimal parameters were trained in the GBM model using the data from the training set, and the simple algorithm for GBM proceeds as follows:

Step 1. Construct a training dataset {*y*_*i*_, *x*_*i*_}_*i*_^*N*^ trained on *N* samples, where *y* is the outcome variable and *x* is the independent variable. The outcome variable *y* was defined as efficacy (classified as poor efficacy and good efficacy), and the independent variable *x* included 14 indicators including age, gender, prominence, and type of prominence.

Step 2. Set initial prediction model

(1) $$\begin{array}{c} F_{0}\left(x\right)=0, \end{array}$$

and residual

(2) $$\begin{array}{c} r_{i}=y_{i}. \end{array}$$

Step 3. For iteration

(3) $$\begin{array}{c} m=1,2,3,\cdots ,M. \end{array}$$

Step 4. The fitting regression tree ${\hat{f}}_{m}$ has *L* endpoints, and the interaction depth is

(4) $$\begin{array}{c} d=L-1. \end{array}$$

Step 5.

(5) $$\begin{array}{c} F_{m}\left(x\right)=F_{m-1}\left(x\right)+\mu {\hat{f}}_{m}\left(x\right). \end{array}$$

Step 6.

(6) $$\begin{array}{c} r_{i}⟵r_{i}-\mu {\hat{f}}_{m}\left(x\right). \end{array}$$

Step 7.

(7) $$\begin{array}{c} F_{M}\left(x\right)=\overset{M}{\underset{m=1}{\sum }}\mu {\hat{f}}_{m}\left(x\right). \end{array}$$

The test set finally validated the predictive model. At the same time, the effects of independent variables on outcome variables were analyzed to find the most critical factors affecting the outcome variables.

### 2.4. Statistical Analysis

The SPSS 23.0 software was used for statistical data analysis. The comparison of success rates of each model was performed using the chi-square test. When the difference was found to be statistically significant by the chi square test, to avoid excessive multiple comparisons to improve the power of the test, the differences among the groups were further analyzed by the pooled cell method. The *t*-test was used to analyze the differences between groups at different times of treatment time. The receiver-operator characteristics curve (ROC) was used to evaluate the sensitivity and specificity of the model.

## 3. Result

### 3.1. Efficacy Analysis

Before treatment, the pain VAS score of 142 patients with lumbar disc herniation in this study was 6.8 (3.0-10.0) points, and the posttreatment pain VAS score was 4.3 (0.1-7.8) points. After physical therapy, the patient's pain was significantly relieved. The symptoms of lumbar disc herniation were also considerably improved by comparing the MRI of the lumbar disc before and after treatment (Figure 1).

### 3.2. Mathematical Expressivity Analysis

The regression curves of each case showed some differences, and the regression curves of some patients showed “S” type characteristics (Figure 2(a)). Some additional patients showed regression lines that resembled straight lines (Figure 2(b)). The coefficient of determination of the 142 patients in this study was 0.731 (0.001-0.979). The global coefficient of determination was 0.721, suggesting that this model can better express the course of physical therapy for patients with lumbar disc herniation.

### 3.3. Effective Case Prediction Power Analysis

The predictive ability of the length of treatment for effective vs. ineffective cases gradually improved with the number of treatment sessions, and specific data are detailed in Table 1. The difference between them was statistically significant by the chi-square test for the data in the table. Their success rates were all predicted to be above 80% based on validity completed with more than five measurements, and they were relatively close to each other. However, the predictions obtained based on 2-4 measurements are relatively close to each other and have low predictive power. After merging the cells, the predicted outcomes of measurements more than 5 times were compared with those of measurements within 4 times, and the difference between them was found to be statistically significant.

### 3.4. Remission Magnitude Predictive Power Analysis

The predictive ability of the remission range of the whole course of treatment varied in different treatment duration. With the increase in treatment times, the difference between the predicted and measured values gradually decreases. The prediction success rate of remission amplitude obtained by each prediction model increases with treatment times (Table 2). The predictive power of 2-4 measurements was low, and all of them had less than 50% correct. The accurate rates of prediction results of 5-7 measurements were all at 60% sufficient, and the accurate rates of 8-9 measurements were relatively high. All of them reached more than 80%.

According to the characteristics of prediction ability, the treatment duration was combined into 2~4 times, 5~7 times, and 8-9 times. It was found that the difference between the groups of 2-4 times and 5-7 times was statistically significant (*P* < 0.01). The difference between the groups of 8-9 times and the group of 5-7 times was also statistically significant (*P* < 0.01).

### 3.5. Prediction Model of Short-Term Prognosis Based on GBM

The optimal parameters of GBM model were obtained through grid search and manual debugging. The final parameters are adjusted to (learning_rate = 0.1, *n*_estimators = 1000, max_depth = 4, min_samples_split = 2, min_samples_leaf = 1, subsample = 1, max_features = ^‘^sqrt′, random_state = 10). The test set data verify the prediction model constructed by the training set. The influencing factors in the GBM model were ranked by importance, and the top five are the sagittal diameter of protrusion, the degeneration level of the surgical segment, age, the time from initial symptom to operation, and the degeneration level of the adjacent segment.

The area under the ROC curve (AUC) of the GBM prediction model was 0.936 [95% CI (0.782, 0.973)]. The sensitivity, specificity, and Youden index were 93.3%, 87.5%, and 0.808, respectively. The AUC of logistic regression analysis was 0.883 [95% CI (0.756, 0.914)]. The sensitivity, specificity, and Youden index were 88.6%, 67.8%, and 0.624, respectively. The prediction effects of the two prediction models were statistically significant (*P* < 0.001) (Figure 3).

## 4. Discussion

Rehabilitation therapy plays an essential role in many treatment fields, including bone and joint system diseases, nervous system diseases, and circulatory and respiratory system diseases [25–27]. From the analysis of treatment purpose, rehabilitation treatment pays more attention to function acquisition. From the comparison of characteristic entropy, rehabilitation treatment means are diverse and targeted, making rehabilitation treatment prescriptions richer and more complex than drug treatment, showing more apparent individualized treatment characteristics [28]. However, it also brings difficulties to efficacy evaluation and prediction. For example, there are a large number of reports on efficacy prediction. Many researchers try to predict the treatment outcome by looking for the relationship between clinical characteristics and functional outcomes. Still, the prediction ability is significantly reduced due to the complexity of patient characteristics and the richness of treatment methods.

In the actual rehabilitation treatment, it is found that the true efficacy of rehabilitation prescription can be understood to a certain extent by observing the patient's treatment feedback information, which can predict the treatment effect [29, 30]. However, how to choose a reasonable length of treatment time so that we can save medical resources to the greatest extent terminates the treatment scheme with poor curative effect in time, accurately predicts the curative effect, and prevents unnecessary prescription adjustment. Thus, we need to have a sufficient understanding of the characteristics of the treatment process. Through the long-term observation of the treatment process, this study proposed to use the logistic curve model and GBM model to predict and analyze the curative effect of physical therapy and nursing of lumbar disc herniation.

In clinical treatment, the remission process of different patients is different. The main difference is the remission speed and onset time [31, 32]. A mathematical model that can fully reflect the above characteristics must be constructed [33–35]. The logistic model is an “S” curve with upper and lower asymptotes. In the model construction, we pay special attention to the parameter design: for example, the characteristics of onset time and descent rate are fully expressed by parameters *a* and *b*. Relevant research shows that GBM has a strong classification ability in many machine learning. GBM is an improved forward learning machine learning enhancement algorithm for regression and classification problems. Its fundamental theory is to produce a prediction model composed of weak learners or essential learners and gradually obtain approximately accurate prediction results from vulnerable learners to solid learners.

From the analysis of mathematical expression ability, the logistic regression model is satisfied with the expression ability of the physical treatment process of lumbar disc herniation. The global determination coefficient is 0.721. In the analysis of the predictive ability of different treatment practice lengths on the efficacy of the whole course of treatment, with the extension of treatment time, both effectiveness prediction and remission amplitude prediction show a good change prediction trend. In the effectiveness prediction analysis, when the forecast is made according to the measured values more than five times (because the pain evaluation is completed before each treatment, that is, more than four experimental treatments), the prediction ability is close. The accuracy rate is stable at more than 80% in the prediction analysis of lumbar disc herniation. When 8-9 measurements are used for prediction in the mitigation amplitude analysis, the accuracy is more than 80%. GBM usually takes the weak prediction model as the benchmark model to generate a complex prediction model. It constructs the model in a phased manner and optimizes it by selecting any differentiable function as the loss function, which can better fit the data. However, there are still some limitations to this study. The sample size of this study was not large enough, which may cause the overfitting of the model. Moreover, the model's prediction accuracy requires the physical therapy process of patients many times, the experimental data are more strictly adopted, and subsequent studies can simplify the model and take a more convenient approach.

## 5. Conclusions

In conclusion, it is feasible and accurate to use the logistic curve model and GBM model to predict rehabilitation treatment's mathematical expression and curative effect for patients with lumbar disc herniation. The treatment effectiveness and remission range can be effectively expected by analyzing more than five measured values obtained from more than four experimental treatments.

## Figures and Tables

**Figure 1:** Comparison of magnetic resonance images before and after physical therapy. Compared with the image before treatment (a), disc herniation (arrow) after treatment (b) decreased significantly.

**Figure 2:** Comparison of regression curves of typical patients. (a) “S” type characteristics. (b) Linear characteristics.

**Figure 3:** ROC curve of GBM model and logistic regression analysis model.

**Table 1:** Analysis of ability to predict curative effect for different treatment duration (cases, %).

Length of treatment	Successful prediction	Unsuccessful prediction
1^st^-2^nd^	87/61.3	55/38.7
1^st^-3^rd^	105/73.9	37/26.1
1^st^-4^th^	110/77.5	32/22.5
1^st^-5^th^	120/84.5	22/15.5
1^st^-6^th^	121/85.2	21/14.8
1^st^-7^th^	114/80.3	28/19.8
1^st^-8^th^	119/83.8	23/16.2
1^st^-9^th^	128/90.1	14/9.9

**Table 2:** Analysis of ability to predict remission amplitude for different treatment time lengths (cases, %).

Length of treatment	Successful prediction	Unsuccessful prediction
1^st^-2^nd^	46/32.4	96/67.6
1^st^-3^rd^	59/41.6	83/58.5
1^st^-4^th^	64/15.1	78/64.9
1^st^-5^th^	93/65.5	49/34.5
1^st^-6^th^	82/57.7	60/42.3
1^st^-7^th^	92/64.8	50/.35.2
1^st^-8^th^	114/80.3	28/19.7
1^st^-9^th^	124/87.3	18/12.7

## Data Availability

The data used to support the findings of this study are available from the corresponding author upon request.

## References

[1] Sınmaz T., Akansel N. (2021). Experience of pain and satisfaction with pain management in patients after a lumbar disc herniation surgery. *Journal of Perianesthesia Nursing*.

[2] Heisinger S., Huber D., Matzner M. P. (2021). Online videos as a source of physiotherapy exercise tutorials for patients with lumbar disc herniation-a quality assessment. *International Journal of Environmental Research and Public Health*.

[3] Hao F. (2021). Analysis of the effect of traction combined with paraffinotherapy on lumbar function in patients with lumbar disc herniation. *American Journal of Translational Research*.

[4] Azimi P., Benzel E. C. (2016). Cut-off value for pain sensitivity questionnaire in predicting surgical success in patients with lumbar disc herniation. *PLoS One*.

[5] Moon S. H., Lee J. I., Cho H. S., Shin J. W., Koh W. U. (2017). Factors for predicting favorable outcome of percutaneous epidural adhesiolysis for lumbar disc herniation. *Pain Research & Management*.

[6] Ostafiński K., Świątnicki W., Szymański J. (2020). Predicting conservative treatment failure in patients with lumbar disc herniation. Single center, case-control study. *Clinical Neurology and Neurosurgery*.

[7] Pedersen C. F., Andersen M., Carreon L. Y., Eiskjær S. (2020). Applied machine learning for spine surgeons: predicting outcome for patients undergoing treatment for lumbar disc herniation using pro data. *Global Spine Journal*.

[8] Wang H., Zhang D., Ma L., Shen Y., Ding W. (2015). Factors predicting patient dissatisfaction 2 years after discectomy for lumbar disc herniation in a Chinese older cohort. *Medicine*.

[9] Yoo B. R., Son S., Lee S. G., Kim W. K., Jung J. M. (2021). Factors predicting the clinical outcome after trans-sacral epiduroscopic laser decompression for lumbar disc herniation. *Neurospine*.

[10] Han M., Liu L., Hu M., Liu G., Li P. (2022). Medical expert and machine learning analysis of lumbar disc herniation based on magnetic resonance imaging. *Computer Methods and Programs in Biomedicine*.

[11] Han Z., Li Z., Liu K., Yan L. (2020). Named data networking with neural networks for intelligent image processing information systems. *Enterprise Information Systems*.

[12] Han Z., Liu K., Li Z., Luo P. (2021). A pre-check operator for reducing algorithmic optimisation time in image processing applications. *Enterprise Information Systems*.

[13] Shi J., Ye Y., Zhu D., Su L., Huang Y., Huang J. (2021). Automatic segmentation of cardiac magnetic resonance images based on multi-input fusion network. *Computer Methods and Programs in Biomedicine*.

[14] Liu Y., Fang Q., Jiang A., Meng Q., Pang G., Deng X. (2021). Texture analysis based on U-Net neural network for intracranial hemorrhage identification predicts early enlargement. *Computer Methods and Programs in Biomedicine*.

[15] Yang Y., Zheng J., Du Z., Li Y., Cai Y. (2021). Accurate prediction of stroke for hypertensive patients based on medical big data and machine learning algorithms: retrospective study. *JMIR Medical Informatics*.

[16] Hu B., Wang C., Jiang K. (2021). Development and validation of a novel diagnostic model for initially clinical diagnosed gastrointestinal stromal tumors using an extreme gradient-boosting machine. *BMC Gastroenterology*.

[17] Kumar S., Singh K. K. (2021). Rain garden infiltration rate modeling using gradient boosting machine and deep learning techniques. *Water Science and Technology*.

[18] Luo Z., Huang F., Liu H. (2020). PM_2.5_ concentration estimation using convolutional neural network and gradient boosting machine. *Journal of Environmental Sciences (China)*.

[19] Mahapatra S., Sahu S. S. (2022). ANOVA‐particle swarm optimization-based feature selection and gradient boosting machine classifier for improved protein-protein interaction prediction. *Proteins*.

[20] Rufo D. D., Debelee T. G., Ibenthal A., Negera W. G. (2021). Diagnosis of diabetes mellitus using gradient boosting machine (lightgbm). *Diagnostics*.

[21] Pilato F., Calandrelli R., Distefano M., Tamburrelli F. C. (2021). Multidimensional assessment of cervical spondylotic myelopathy patients. Usefulness of a comprehensive score system. *Neurological Sciences*.

[22] Gong L., Ma H. N., Yi P., Tan M. S. (2021). Flexion dysfunction of atlanto-occipital joint associated with cervical spondylosis. *Orthopaedic Surgery*.

[23] Therriault T., Rospert A., Selhorst M., Fischer A. (2020). Development of a preliminary multivariable diagnostic prediction model for identifying active spondylolysis in young athletes with low back pain. *Physical Therapy in Sport*.

[24] Kelly A. M. (2001). The minimum clinically significant difference in visual analogue scale pain score does not differ with severity of pain. *Emergency Medicine Journal*.

[25] Arai M. (2021). Evaluating the usefulness of *Ninjin'yoeito Kampo* medicine in combination with rehabilitation therapy in patients with frailty complicated by intractable dizziness. *Neuropeptides*.

[26] Lou H., Li Z., Pang T. (2021). Electrocupuncture combined rehabilitation therapy for upper limb spasticity after stroke. *Medicine*.

[27] Tsukagoshi M., Harimoto N., Araki K. (2021). Impact of preoperative nutritional support and rehabilitation therapy in patients undergoing pancreaticoduodenectomy. *International Journal of Clinical Oncology*.

[28] Langhorne P., Bernhardt J., Kwakkel G. (2011). Stroke rehabilitation. *The Lancet*.

[29] Van Stan J. H., Whyte J., Duffy J. R. (2021). Rehabilitation treatment specification system: methodology to identify and describe unique targets and ingredients. *Archives of Physical Medicine and Rehabilitation*.

[30] Whyte J., Dijkers M. P., Hart T. (2019). The importance of voluntary behavior in rehabilitation treatment and outcomes. *Archives of Physical Medicine and Rehabilitation*.

[31] Gassert R., Dietz V. (2018). Rehabilitation robots for the treatment of sensorimotor deficits: a neurophysiological perspective. *Journal of Neuroengineering and Rehabilitation*.

[32] Tijsen L. M., Derksen E. W., Achterberg W. P., Buijck B. I. (2019). Challenging rehabilitation environment for older patients. *Clinical Interventions in Aging*.

[33] Formanowicz D., Krawczyk J. B., Perek B., Lipski D., Tykarski A. (2021). Management of high-risk atherosclerotic patients by statins may be supported by logistic model of intima-media thickening. *Journal of Clinical Medicine*.

[34] Guo Z., Meng L., Tian S. (2021). A five-parameter logistic model to predict the possibility of misdiagnosis for improving the specificity of lugol chromoendoscopy in the diagnosis of esophageal neoplastic lesions. *Frontiers in Oncology*.

[35] Jeong S., Luo G., Gao Q. (2021). A combined cox and logistic model provides accurate predictive performance in estimation of time-dependent probabilities for recurrence of intrahepatic cholangiocarcinoma after resection. *Hepatobiliary Surgery and Nutrition*.

